# A Systematic Review and Meta-Analysis on Randomized Control Trials for Preoperative Rehabilitation in Patients Planning for Joint Replacement Surgery for Better Outcomes

**DOI:** 10.1155/2022/4287555

**Published:** 2022-03-10

**Authors:** Haibo Yin, Bin Chen, Zhu Xu

**Affiliations:** The Second Affiliated Hospital, Jiaxing University, Jiaxing, China

## Abstract

**Background:**

The clinical influence of the preoperative and postoperative therapies for recovery after the joint replacement surgery is still questionable. This study of systematic review and meta-analysis focuses on analyzing the clinical effects of preoperative rehabilitation among the patients who are planning to opt for joint replacement surgery for enhanced results.

**Objective:**

Randomized clinical trials were selected where preoperative therapeutic exercises were performed by adults for preoperative rehabilitation in patients who were planning for replacement surgery for better outcomes and identified through databases and screening. Two reviewers were responsible for extracting appropriate studies, relevant data, assessing the risks, therapeutic validity, etc. *Material and Methods*. We performed random-effects meta-analysis for calculation of risk ratios and odds ratios, for knee and hip surgery cases. Analysis of length of hospital stay, short-term-based recovery period during hospital stay, total hip replacement functional recovery during hospital stay, short-term recovery of self-reported functioning, etc. was performed.

**Results:**

Functional scores, postoperative pain, recovery time, length of hospital stay, and quality of life were studied. Of the seven studies included, the data of 614 patients were studied. The total number of participants in both exercise and control groups was analyzed to assess the bias of the study where the risk ratio was 0.96 and (0.74–1.25) was the 95% CI. Short-term-based recovery period during hospital stay for knee replacement was analyzed where 0.87 was the risk ratio and (0.61–1.23) was the 95% CI and for hip replacement where 0.99 was the risk ratio and (0.68–1.44) was the 95% CI. The RR for total hip replacement functional recovery during hospital stay was 0.80 with 95% CI (0.54–1.19). The RR for short-term recovery of self-reported functioning was 0.98 with 95% CI (0.76–1.26). Outcome analysis for pain and functionality evaluation was performed and assessed using WOMAC, HOOS, and HHS scores where the standardized mean difference was 0.38 and (0.20–0.57) was the 95% CI in hip surgery pain analysis and in knee surgery, 0.00 was the standardized mean difference and (−0.18–0.19) was the 95% CI.

**Conclusion:**

Long-term outcomes were not affected by the preoperative rehabilitation. Though there was a slight improvement in early postoperative pain, this is not much of clinical significance.

## 1. Introduction

The total joint replacement surgery is observed as one of the most efficient medical arbitrations which leads to consequential relief from pain and refines the physical function and life conditions for the patients who suffer from critical osteoarthritis [1]. Although the rehabilitation for a remarkable number of patients remains tough and extends, many of them never experience the effectiveness post operation [2, 3]. Thus, the policymakers, experimenters, and clinicians are still performing research studies for better ways to enhance the duration of recovery for the patients going through the total joint replacement. The total knee arthroplasty (TKA) is a voluntary surgical approach post the failure of conventional administration among the patients going through the improved knee osteoarthritis (KOA) [4].

Many times severe knee osteoarthritis is accompanied by recurrent pain, limited joint flexibility, quadriceps femoris weakness, and decreased function in activities of daily living related to exercise [5, 6]. However, the level of pain and the flexibility of joints are enhanced post surgery, and 20–30% are unsatisfied with the outcomes [7]. The occurrence of infection linked with these kinds of replacements has been predicted to be anyplace from 0.39% to 2.5% for key total knee arthroplasty [8]. Throughout the preoperative standby time, the flexibility of joints and the level of pain become worse, along with which the muscles neighboring the joint section further leads to atrophy because of the diminished assistance and the neuromuscular obstruction [6]. As seen in the outcome, the contribution in the activities of the daily living and the degree of physical activity (PA) worsens [9].

In this study, we have performed an updated methodological systematic review along with meta-analysis to elucidate the supporting evidence for preoperative rehabilitation among the patients opting for joint replacement surgery.

## 2. Material and Methods

### 2.1. The Study Selection

In this research study, the patients, involvement, resource-related outcomes, and length of hospital stay along with readmission were taken into consideration. We explored the electronic databases to extract the applicable studies such as the PubMed, Cochrane Central Register of Control Trials, CINAHL, and Embase from the period 2006 to 2020. These eligible research studies included should meet the following criteria: (i) randomized control trials, (ii) comparators including preoperative vs. postoperative rehabilitation programs and control vs. training group, (iv) outcomes, and (v) language of the studies included English.

### 2.2. Search Approach

We performed the Preferred Reporting Items for Systematic Reviews and Meta-Analysis (PRISMA) and defined the research-based questionnaire to discover the related research studies. The keywords used for the search were “pre-operative rehabilitation,” “joint replacement surgery,” “rehabilitation,” “knee osteoarthritis,” “hip replacement,” “knee replacement,” “kinesiotherapy,” “joint replacement,” “physiotherapy,” “physical therapy,” “hydrotherapy,” “randomized,” “randomized controlled trial,” “randomized controlled trial,” and “randomized controlled trial.”

### 2.3. Inclusion and Exclusion Criteria

A total of 205 studies were identified to be relevant from the search through relevant set of keywords along with 4 additionally identified records. Out of this total 209 research studies, 104 studies were identified to be relevant as per the aim of this study, and remaining 97 studies were rejected due to the following exclusion criteria: insufficient patient data, nonclinical studies, no postoperative data, no outcome of interest, non-RCTs, review paper, abstracts, letters, or editorials. Finally, 7 research studies were observed eligible for systematic review and meta-analysis based on inclusion criteria. Among these 7 research studies, two of them included were about the patient going through total knee replacement, other three were about total hip replacement, and the remaining two were either hip or knee replacement (Table 1).

### 2.4. Observation Indicators

The MLR and NLR were tested for relationships with AKI development and prognosis using multivariable logistic regression, with the results presented as odds ratios (ORs). The predictive usefulness of the MLR and NLR for the development of AKI and in-hospital mortality was evaluated using receiver operating curves (ROC).

### 2.5. Statistical Analysis

Variables were shown as medians with interquartile ranges in continuous data, while categorical variables were shown as frequency counts in categorical data. For both categorical and continuous data, the chi-square test was used to make comparisons between groups. The MLR's relationship with other factors was investigated using Spearman's correlation. The Youden index was used to calculate cut-off values as well as the sensitivity and specificity for parameters. For all of the studies, a two-tailed p>0.05 indicated statistically significant. SPSS 16 (Chicago, IL, USA) was used to conduct the entire data study.

## 3. Result

### 3.1. The Forest and Funnel Plot of Short-Term-Based Recovery Period during Hospital Stay for Knee Replacement

Analysis for short-term-based recovery period during hospital stay for knee replacement was performed where the risk ratio was 0.87 and (0.61–1.23) was the 95% CI (Figure 1). The forest plot of short-term-based recovery period during hospital stay for knee replacement is shown in Figure 2, and the funnel plot for the same study is shown in Figure 3. Short-term-based recovery period duration during hospital stay for hip replacement analysis was performed where the risk ratio is 0.99 and (0.68–1.44) is the 95% CI. The forest and funnel plots for this analysis are shown in Figure 4 and 5, respectively. Short-term-based recovery period during hospital stay is recorded in Table 2. The total number of participants in both exercise and control groups was analyzed to assess the bias of study where 0.96 was the odds ratio and (0.74–1.25) was the 95% CI. The forest plot and funnel plots are shown in Figure 6 and 7, respectively.

### 3.2. The Forest and Funnel Plot of Total Hip Replacement Functional Recovery

The risk ratio of total hip replacement functional recovery during hospital stay was 0.80 with 95% CI (0.54–1.19). The forest plot for the same is shown in Figure 8, and the funnel plot is shown in Figure 9. The risk ratio for short-term recovery of self-reported functioning was 0.98 with 95% CI (0.76–1.26), forest plot for short-term recovery is shown in Figure 10, and funnel plot is shown in Figure 11.  Table 3 presents the outcome score for pain evaluation (postoperative) hip and knee surgery. Outcome score analysis using WOMAC: Western Ontario MacMaster, HOOS: Hip Disability and Osteoarthritis Outcome Score, and HHS: Harris Hip Score for pain evaluation (postoperative) of hip and knee surgery was performed where the standardized mean difference was 0.38 and (0.20–0.57) was the 95% CI in hip surgery pain analysis, and 0.00 was the standardized mean difference and (−0.18–0.19) was the 95% CI in knee surgery. No significant changes were observed (Figures 12 and 13).  Figure 14 shows an overview of the methodological quality results.

## 4. Discussion

The enhanced recovery after surgery (ERAS) has expeditiously been recognized by the anesthetists. The preoperative programs assimilating the multimodal, proof-related involvement are identified as fast-track or ERAS pathways [16]. The enhanced revival post surgery constitutes the next step in the process of evolution of regulated care. In the evaluation of elements to the deficient physical as well as cognitive operation post total hip or knee arthroplasty, important ERAS ideas were being successfully implemented to the elective joint arthroplasty. Therefore, the future performance is guided towards regulating the stress-related response in the course of instant recovery and optimizing postdischarge purpose. For high-level knee osteoarthritis patients, total knee arthroplasty (TKA) is the usual surgical procedure [17].

This guides to a higher level of patient contentment as there are substantial medium to long-term comforts which comprises of the development in the quality of life and relieve from pain along with the recovery function. However, the total knee arthroplasty develops certain complications such postoperative soreness, restricted functions of joints, and the analgesia-based harmful effects that expend a huge outcome on the postoperative rehabilitation [18].

The results of the study have demonstrated that the patients who underwent preoperative rehabilitation using trainings and exercises prior to joint replacement surgeries were too small to be significant clinically. Hence pre-habilitation produced a very significant effect on postoperative pain and functionality scores, patient recovery, length of stay, and other crucial factors. Therefore, future research must focus on measuring more clinically significant outcomes in the randomized trails which will be of importance to be documented and analyzed for effective evaluation between the two groups. No significant benefit of the therapeutic exercises or training was documented; hence, other clinical factors must also be measured in studies to analyze the outcomes critically.

## 5. Conclusion

The evidence suggests that pre-habilitation has very slight evidence of improvement in the functioning of a person, recovery time, recovery efficiency, function among patients, postoperative pain, who underwent knee or hip joint replacement surgery. The effects were for a short term, but they were not significant clinically. Long-term outcomes such as quality of life and length of stay were not affected by the preoperative rehabilitation. Though there was slight improvement in early postoperative pain, this is not much of clinical significance. For the sake of therapeutic validity, the studies must be significantly documented for more clinically significant parameters for critical analysis of the outcomes of training.

## Figures and Tables

**Figure 1:** PRISMA study over the study methods.

**Figure 2:** Forest plot for short-term-based recovery period during hospital stay for knee replacement.

**Figure 3:** Funnel plot for short-term-based recovery period during hospital stay for knee replacement.

**Figure 4:** Forest plot for short-term-based recovery period during hospital stay for hip replacement.

**Figure 5:** Funnel plot for short-term-based recovery period during hospital stay for hip replacement.

**Figure 6:** Forest plot for number of participants in exercise and control groups.

**Figure 7:** Funnel plot for number of participants in exercise and control groups.

**Figure 8:** Forest plot for total hip replacement functional recovery during hospital stay.

**Figure 9:** Funnel plot for total hip replacement functional recovery during hospital stay.

**Figure 10:** Forest plot for short-term recovery of self-reported functioning.

**Figure 11:** Funnel plot for short-term recovery of self-reported functioning.

**Figure 12:** Forest plot for outcome score for postoperative pain evaluation in hip surgery.

**Figure 13:** Forest plot for outcome score for postoperative pain evaluation in knee surgery.

**Figure 14:** Risk of bias and applicability concerns summary.

**Table 1:** Characteristics of the studies included.

Characteristics	[10]	[11]	[6]	[12]	[13]	[14]	[15]
Study location	The Netherlands	Italy	USA	Italy	Turkey	Australia	United Kingdom
Mean age	76	63.4	67.0	66.5	51.3	69.7	69.8
Number of patients	21	23	108	122	60	160	120
Women, n (%)	66	60.8	54	48	35.5	78.9	52.9
Trial design	Randomized controlled trial	Randomized controlled trial	Randomized controlled trial	Randomized controlled trial	Randomized controlled trial	Randomized controlled trial	Randomized controlled trial
Type of surgery	Total hip replacement	Total hip replacement	Total hip replacement/total knee replacement	Total knee replacement	Total hip replacement	Total knee replacement	Total knee replacement
Type of exercise	Functional exercise	Resistance exercise	Resistance exercise	Preoperative home exercise	Resistance exercise	Stretching warm-up training	Resistance exercise
BMI	31.6	NR	34.8	28.5	NR	27.4	32.7

NR, not reported.

**Table 2:** Short-term-based recovery period during hospital stay.

Characteristics	Groups	[10]	[11]	[6]	[12]	[13]	[14]	[15]
Number of participants	Exercise group	10	11	32	61	30	18	60
	Control group	11	12	31	61	30	20	61
Short-term-based recovery period during hospital stay	Training (knee replacement)	8	N/A	14	N/A	N/A	N/A	23
	Control (knee replacement)	9	N/A	15	N/A	N/A	N/A	29
	Training (hip replacement)	N/A	11	25	N/A	N/A	N/A	N/A
	Control (hip replacement)	N/A	12	24	N/A	N/A	N/A	N/A
Total hip replacement functional recovery during hospital stay	Intervention	8	N/A	20	N/A	N/A	N/A	N/A
	Control	9	N/A	26	N/A	N/A	N/A	N/A
Short-term recovery of self-reported functioning	Intervention	N/A	11	25	N/A	29	N/A	N/A
	Control	N/A	12	24	N/A	30	N/A	N/A
Participants	Total	21	23	108	122	60	160	120

**Table 3:** Outcome score for pain evaluation (postoperative) hip and knee surgery.

Pain score	[10] (HOOS pain; hip surgery)	[11] WOMAC pain (hip surgery)	[6] WOMAC (hip surgery)	[6] WOMAC (knee surgery)	[12] (knee surgery)	[13] HHS (hip surgery)	[14] (WOMAC score) knee	Reference [15] (WOMAC); knee
Exercise group	55.3 ± 12.0	8.0 ± 3.8	7.5 ± 3.0	7.0 ± 2.0	53 ± 29	64.46 + 6.92	0.98 ± 0.99	26 ± 17.7
Control group	49.3 ± 17.0	11.0 ± 3.6	8.5 ± 3.0	6.5 ± 4.5	55 ± 27	59.36 + 6.82	1.3 ± 1.1	24.6 ± 16.8
Total	100	20	20	20	100	100	10	100

WOMAC: Western Ontario MacMaster; HOOS: Hip Disability and Osteoarthritis Outcome Score; HHS: Harris Hip Score.

## Data Availability

The data used to support this study are available from the corresponding author upon request.
